The article "Comparison of Presurgical Dental Models Manufactured with Two Different Three-Dimensional Printing Techniques" was published in 2020. Journal: J Healthc Eng.

# Comparison of Presurgical Dental Models Manufactured with Two Different Three-Dimensional Printing Techniques

**DOI:** 10.1155/2020/8893338

**Published:** 2020-09-29

**Authors:** Marcin Metlerski, Katarzyna Grocholewicz, Aleksandra Jaroń, Mariusz Lipski, Grzegorz Trybek

**Affiliations:** ^1^Department of Oral Surgery, Pomeranian Medical University in Szczecin, Al. Powstańców Wlkp. 72, 70-111 Szczecin, Poland; ^2^Department of Interdyscyplinary Dentistry, Pomeranian Medical University in Szczecin, Al. Powstańców Wlkp. 72, 70-111 Szczecin, Poland; ^3^Department of Preclinical Conservative Dentistry and Preclinical Endodontics, Pomeranian Medical University in Szczecin, Al. Powstańców Wlkp. 72, 70-111 Szczecin, Poland

## Abstract

Three-dimensional printing is a rapidly developing area of technology and manufacturing in the field of oral surgery. The aim of this study was comparison of presurgical models made by two different types of three-dimensional (3D) printing technology. Digital reference models were printed 10 times using fused deposition modelling (FDM) and digital light processing (DLP) techniques. All 3D printed models were scanned using a technical scanner. The trueness, linear measurements, and printing time were evaluated. The diagnostic models were compared with the reference models using linear and mean deviation for trueness measurements with computer software. Paired *t*-tests were performed to compare the two types of 3D printing technology. A *P* value < 0.05 was considered statistically significant. For FDM printing, all average distances between the reference points were smaller than the corresponding distances measured on the reference model. For the DLP models, the average distances in the three measurements were smaller than the original. Only one average distance measurement was greater. The mean deviation for trueness was 0.1775 mm for the FDM group and 0.0861 mm for the DLP group. Mean printing time for a single model was 517.6 minutes in FDM technology and 285.3 minutes in DLP. This study confirms that presurgical models manufactured with FDM and DLP technologies are usable in oral surgery. Our findings will facilitate clinical decision-making regarding the best 3D printing technology to use when planning a surgical procedure.

## 1. Introduction

Three-dimensional (3D) printing is a rapidly developing area of technology and manufacturing in the field of oral surgery and is playing a meaningful role in diagnosis, surgical planning, implants, training before surgery, and education [1, 2]. Printed models can help overcome some of the operative difficulties encountered, including surgical resection of periapical tooth lesions, sinus augmentation, and autotransplantation [3–5].

Three-dimensional printed models could also be used as part of the surgical implant guides used for preoperative planning and training. Deeb et al. devised an implant guide by rapid prototyping for clinical use that was found to reduce the time spent on correct implant placement convenience and to improve cost-effectiveness [6]. Templates based on medical models significantly improve the efficiency of the surgical procedure. Use of medical models reduces the risk of surgery failure to 25% and combined use of a medical model and a template reduces the error rate to 5%–10% [7].

Three-dimensional printing based on 3D computed tomography or intraoral scanning data can be used to produce a physical model. The intraoral surface data and radiographic 3D data can be fused, and a procedure that includes a virtual implant planning process and a production implant drilling guide can facilitate dental implantology [8].

A replica graft tooth can be used in autotransplantation surgery. Application of 3D printing technology simplifies the medical procedure and shortens the operating time. Furthermore, use of a rapid prototyping model reduces damage to a donor tooth during preparation of a recipient site [9, 10].

Virtual surgical planning using 3D printing technology also improves the efficiency and surgical precision and shortens work time. Applying this innovative technology enables reconstruction of a nonstandard bone defect. Moreover, application of a printed presurgical model makes it possible to measure the bone defect preoperatively and allows the surgeon to remove a small portion of the bone. The bone graft can be fitted perfectly and fewer screws are needed for stability [11]. Three-dimensional printed objects are used in maxillofacial surgery, usually to make a surgical guide (59%) or an anatomic model (34%) [12].

The 3D printers available on the market use a variety of printing techniques, the most common of which are based on fused deposition modelling (FDM) [13]. FDM was the first thermoplastic technology used in “home” printers. Using this method, thermoplastic material is extruded through a nozzle onto a build platform. However, models produced by this technology are characterized by high porosity and variable mechanical strength [14, 15].

Another technique used in 3D printing is digital light processing (DLP), which uses a light-cured resin technique in which the resin is cured with a projector light source. The aim is to build a model upside down on the platform. Such models have good accuracy and create a smooth surface. Both FDM and DLP 3D printing technologies are of low cost [15, 16], and in both DLP and FDM technologies, 3D models are created by depositing materials layer by layer in an additive manufacturing process [14, 16].

The applications of 3D printing are increasing in dental surgery [17], where 3D printed models are most often used to create surgical templates and diagnostic models [6, 13, 15]. There are a lot of studies comparing orthodontic models with production technology [18]. There has been no study comparing different 3D printing technologies available for creating presurgical models.

The aim of this study was to compare presurgical models created using two different types of 3D printing technology. The null hypothesis was that there would be no significant difference in trueness between the printed presurgical models.

## 2. Materials and Methods

A monocentric study was conducted on 10 patients in whom an implantation procedure was planned. The exclusion criteria were toothlessness and the necessity to carry out augmentation procedure before the implantation. All procedures were conducted after obtaining the approval of the Ethics Committee of Pomeranian Medical University, Poland (KB-0012/483/11/16). Clinicians participating in the study use an intraoral scanner and 3D printing in everyday practice, and they are distinguished by extensive experience in the use of intraoral scanners. The study methodology is shown in Figure 1.

Dental arch was scanned for each patient using a TRIOS 3 intraoral scanner (3Shape, Copenhagen, Denmark). Third molars were not included. The 3D surface datasets obtained were then digitally converted to orthodontic models using an Ortho Analyzer (3Shape). All scans were saved as stereolithography (stl) files. The model was manipulated using 3D software for working with triangle mesh (Meshmixer, version 3.4.35; Autodesk, San Rafael, CA, USA) to standardize the measurements. Four half-ball indices (diameter, 2.0 mm) were placed on all the models as reference points. The reference points are placed on the basis of the model. The positions of reference points corresponding to central incisors and right and left first molar teeth are shown in Figure 2.

The reference points were linked to the anatomical point and placed on the base because of the missing teeth that were found in the patients. This made it possible to select the same point in different patients.

Digital reference models were printed 10 times each using DLP (Planmeca Creo; Planmeca, Helsinki, Finland) and FDM techniques (see Figure 3) (Zortrax M200; Zortrax, Olsztyn, Poland) as shown in Figure 4.

The DLP models are made of biocompatible light-sensitive resin. In FDM technology, the ABS (acrylonitrile-butadiene-styrene copolymer) material was used. The thickness of the printing layer was 0.05 mm in the DLP group and 0.09 mm in the FDM group; these were the smallest thickness values that could be achieved. All 3D printed models were scanned using an Optical 3D Scanner Activity 855 (KaVo Dental GmbH, Biberach, Germany). All scanned files were saved in stl format. The 3D diagnostic models in the DLP and FDM groups were compared with the reference models. The reference stl models were obtained by scanning the dental arches of the study participants using an intraoral scanner. Determination of reference points allowed superimposition of reference and diagnostic models and calculations. All measurements were performed in the 3D inspection program (GOM Inspect 2018; GOM, Braunschweig, Germany).

The diagnostic models were superimposed on the reference models. Using the abovementioned software, the reference points were manually determined on the highest tip of the half ball by two independent observers (K. G. and M. M.). All measurements were calculated automatically in the GOM Inspect software.

Linear measurements were taken between the tips of the half-ball reference points, 1-2, 2-3, 3-4, and 1-4, respectively (see Figure 2). The measurements were taken by two independent researchers (M. M. and A. J.). In order to minimize random error, all measurement points are described and marked on the models. After selecting the measurement points, the program automatically calculated the distances. The mean deviation for trueness was automatically measured when the diagnostic models from each group were superimposed on the reference models using reference points. Trueness was measured by superimposing the diagnostic models with the corresponding reference models. The mean deviation was an absolute value and represented the best possible match between the diagnostic models to reference models. Endless points forming the diagnostic model have been compared with a reference model. GOM Inspect software delivers colour maps of the mean deviation for trueness with a deviation of up to 0.5 mm (see Figure 4).

### 2.1. Statistical Analysis

Normality was checked using the Shapiro–Wilk test, which showed that study variables follow normal distribution. Paired *t*-tests were performed to determine the trueness of each of the two types of 3D printing technique and to compare the reference model with the diagnostic models. All statistical analyses were performed using SPSS version 24.0 software (IBM. Corp., Warsaw, Poland). The level of statistical significance was set at *P* < 0.05.

## 3. Results

Figure 5 presents the average difference between the linear measurements on FDM and DLP models and the reference model.

For FDM printing, all average distances between the reference points were smaller than the corresponding distances measured on the reference model.

For DLP printing, the average distances in the three measurements were smaller than the original distances (only one average distance measurement was greater). For the distances in points 3-4, a statistically significant difference was found between the studied printing techniques. No statistically significant differences were found for distances at other measurement points.

Figure 6 shows the average trueness deviation measurements for the FDM and DLP models in relation to the reference models. The average of the trueness measurements and printing time with standard deviation is presented in Table 1.

The mean trueness deviation measurement for the DLP replicas was 0.0914 mm smaller than that of the FDM replicas; the difference was statistically significant. Mean printing time for a single model is 285.3 minutes for DLP and 517.6 minutes for FDM technology. Colour maps for trueness images are shown in Figure 4.

## 4. Discussion

The trueness of models created with 3D printers depends on the printing technology used. Each of the technologies available has their advantages and disadvantages. All models manufactured using 3D printing technology have the advantages of a low fracture risk and low weight [19] and ease of data storage and transmission [20]. However, the disadvantages of rapid prototyping methods include the high cost of the printers and printing materials. It is also necessary to have experience in preparing the print materials because the polymers used for printing with the DLP technology are toxic and may be prematurely polymerized [21].

The thickness of the layers of material used for printing determines the accuracy and surface finish of the models. Thicker layers are reportedly less accurate [22]. Although the print layer used in the FDM method (0.09 mm) is thicker than the layer used in the DLP method (0.05 mm), the average print time of a model in the FDM method is longer (see Table 1). Both printers were set to their most accurate settings because the materials accumulate layer by layer in a linear manner. In the case of DLP technology, the whole layer is polymerized at the same time. The results in Table 1 confirm to some extent the earlier reports that manufacturing objects using 3D printing techniques can be fast and efficient [23].

The final product created by a rapid prototyping process will be influenced by the technique used. Printed models are different from virtual objects because of shrinkage of the model during printing [24] and postcuring and the minimal thickness of the layers [25]. Inaccuracies and distortions can be caused by converting and formatting data to an stl file [24]. All these factors could affect the accuracy of the models.

Mean deviations within the limit of 0.3 mm are considered acceptable for diagnostic models [21, 26, 27]. In this study, all the mean deviations of trueness measured for both printing techniques were lower than the acceptable limit (see Figure 6). Furthermore, in general, DLP models had more green areas than the FDM model (see Figure 4). This result can be explained by the differences in the thickness of the layers when building the models.

Models manufactured using 3D printing technology provide important information that is useful in the diagnostic, therapeutic, and educational processes [25] and reduce the risk of surgery failure to 25% [7].

This study is an early attempt to evaluate the accuracy of presurgical models made by two different types of 3D printing technology. This study will facilitate clinical decision-making regarding the best choice of 3D printing technology to use when planning a surgical procedure. To our knowledge, this is the first study to report the accuracy of presurgical models made by two different types of 3D printing technology. Future studies should evaluate other 3D printing methods with different 3D printing machines and materials.

## 5. Conclusions

Within the limitations of this in vitro study, we conclude that presurgical models manufactured with FDM and DLP technologies are usable in oral surgery. Although the differences between the diagnostic and reference models constructed with FDM and DLP technologies were statistically significant, the DLP technique appears to be more precise than the FDM technique.

## Figures and Tables

**Figure 1:** Study methodology.

**Figure 2:** The model with half-ball indices and reference points.

**Figure 3:** Three-dimensional printed models. (a) FDM model. (b) DLP model.

**Figure 4:** Colour maps of the mean deviation for trueness.

**Figure 5:** Linear measurements between reference points.

**Figure 6:** Mean deviation for trueness measurements.

**Table 1:** Average and standard deviation of the trueness measurements and printing time.

Printer technique	Trueness	Time (minutes)
	Mean ± SD	Mean ± SD
FDM (0.09 mm)	0.17 ± 0.024	517.6 ± 62.58
DLP (0.05 mm)	0.08 ± 0.009	285.3 ± 18.38

## Data Availability

Linear measurement data are available upon request to the corresponding author.
